RETRACTED

# Application of Deep Reinforcement Learning Algorithm in Uncertain Logistics Transportation Scheduling

**DOI:** 10.1155/2021/5672227

**Published:** 2021-09-25

**Authors:** Yunmei Yuan, Hongyu Li, Lili Ji

**Affiliations:** School of Nanjing Institute of Railway Technology, Nanjing, Jiangsu 210031, China

## Abstract

Nowadays, finding the optimal route for vehicles through online vehicle path planning is one of the main problems that the logistics industry needs to solve. Due to the uncertainty of the transportation system, especially the last-mile delivery problem of small packages in uncertain logistics transportation, the calculation of logistics vehicle routing planning becomes more complex than before. Most of the existing solutions are less applied to new technologies such as machine learning, and most of them use a heuristic algorithm. This kind of solution not only needs to set a lot of constraints but also requires much calculation time in the logistics network with high demand density. To design the uncertain logistics transportation path with minimum time, this paper proposes a new optimization strategy based on deep reinforcement learning that converts the uncertain online logistics routing problems into vehicle path planning problems and designs an embedded pointer network for obtaining the optimal solution. Considering the long time to solve the neural network, it is unrealistic to train parameters through supervised data. This article uses an unsupervised method to train the parameters. Because the process of parameter training is offline, this strategy can avoid the high delay. Through the simulation part, it is not difficult to see that the strategy proposed in this paper will effectively solve the uncertain logistics scheduling problem under the limited computing time, and it is significantly better than other strategies. Compared with traditional mathematical procedures, the algorithm proposed in this paper can reduce the driving distance by 60.71%. In addition, this paper also studies the impact of some key parameters on the effect of the program.

## 1. Introduction

An intelligent transportation system (ITS) is crucial to the realization of the goal of a smart city [1–4]. With advanced sensing, computing, and communication technologies, intelligent transportation system has gradually become a solution with broad application prospects [5]. Electric vehicle (EV) is currently an environmentally friendly vehicle, rather than internal combustion engines driven by fossil fuels, which can effectively reduce carbon emissions in the process of transportation. Recent academic research and industry surveys show that electric vehicles will bring a revolution to the logistics ecological chain in the near future [6–9].

RETRACTED

In addition, due to the surge of e-commerce demand in recent years, the last-mile distribution of small parcels in ground transportation is becoming an increasingly important burden of the modern transportation system [10]. It is expected that in the mature market, the package delivery market will grow at an annual rate of 7%–10%, while in the developing market, such as China and India, it will grow at a rate of more than 300%. The demand for logistics continues to grow with customers' desire for low-cost and fast logistics services. People are increasingly eager for logistics services with low prices and fast delivery speeds. This brings challenges to it. It is necessary to develop a cost-effective package delivery solution [11] to meet a large number of demands on faster traffic.

Considering the scale, growth, and cost awareness of its technology, it provides a sufficient foundation for the future development of small package last-mile distribution. Many research efforts are devoted to designing new logistics planning solutions to solve increasingly difficult problems [12–14]. For example, an automatic vehicle logistics system (AVLS) is recently proposed, which uses automatic vehicles (AVS) as the logistics carrier [15–17]. AVLS also has the characteristics of unmanned driving and low carbon emissions, which can reduce operating costs while protecting the environment [18]. In addition, the system also brings other benefits for a larger intelligent city environment.

Although the existing research can solve the problem of responding to a large number of logistics requests in a short time, the delay is usually longer in an uncertain logistics transportation system on a city scale. In this way, the smart city in the future is difficult to achieve fast door-to-door delivery, and the system can not adapt to the change and update online information in time [19]. The main reason for this problem is that the logistics carrier has too much computational complexity in calculating the optimal path, which is usually affected by vehicle routing problems (VRPs) and its derivative problems. In a survey on urban VRP, it can be seen that most researchers model the logistics vehicle routing problem as a mixed-integer program (mixed-integer program, MIP). MIP is NP-hard. Although the existing solutions can solve this problem, the scale of the cases studied is usually small [20–22]. In the uncertain logistics transportation scheduling problem of city scale, the calculation time will increase exponentially. This problem is not only related to the last-mile delivery of small packages in electric vehicles but also related to all time-sensitive VRP applications [23, 24]. In order to make full use of the advantages of the modern intelligent transportation system, the intelligent city needs a new online strategy to plan the vehicle route in uncertain logistics transportation with the least calculation time [25, 26].

RETRACTED

At present, there are many scholars who study the problem of random demand vehicle routing: some researchers consider the problem of vehicle routing with random demand, give an overview of this problem, and study various solutions. The concepts and main problems and some attributes of the best solutions are reviewed. Then a new problem-solving framework using the Markov decision-making process is proposed [27]. Some researchers have established a variety of chance-constrained model pairs and random VRP in different situations in response to the problem that the introduction of random factors into the classic path problem may change the structure of these problems [28]. There are also researchers who consider vehicles with limited capacity, driver compensation, and the number of vehicles to optimize the complete itinerary, and subject to many constraints such as time window and vehicle capacity, aiming at the smallest driving distance, combining two types of targets [29]. The researchers used Monte Carlo simulations to obtain an estimate of the reliability of each a priori solution, the possibility that there is no vehicle empty before completing the transportation route, and the expectations related to correcting the route choice behavior after the vehicle is empty before completing the route cost [30]. In this way, an estimate of the expected total cost of different routing options can be obtained. Aiming at the vehicle routing problem with random demand and time window, the researchers, respectively, aim at the lowest expected total cost, maximize on-time delivery and consider the first two at the same time, and propose three probability models to solve the on-time delivery problem from different perspectives [31, 32]. The Rollout algorithm designed in the related literature can effectively solve such problems, reducing the running time by estimating the expected cost of the route.

Generally speaking, for uncertain logistics transportation scheduling problems, the solution methods are similar to deterministic logistics transportation scheduling problems, mainly including genetic algorithm, ant colony algorithm, particle swarm algorithm, and simulated annealing algorithm, as well as the combination and improvement of these algorithms. However, these algorithms cannot handle the uncertainty constraints well. The deep reinforcement learning algorithm in machine learning is more suitable for solving uncertain and exploratory problems, but it has not been widely applied to uncertain logistics and transportation scheduling problems, so it is a good research direction. Therefore, this article proposes a path planning scheme based on deep reinforcement learning technology to solve the problem of uncertain logistics. In addition, due to the short computation time of constructing model training cases based on the optimization method, this paper proposes a Deep Reinforcement Learning (DRL) method to solve the key parameters in the model. This solution is suitable for solving large-scale vehicle routing problems because the speed of path planning using this strategy is very fast. Although the debugging process of model parameters is complicated, this process can be done offline. In addition, unlike the similar training of individual models for each problem instance in the optimization based strategy, this method can deal with related problems well because they follow similar traffic network characteristics. Therefore, the trained model can deal with the uncertain logistics transportation scheduling problem, and the efficiency is much higher than the traditional repeated solution.

RETRACTED

## 2. Uncertain Logistics Transportation System Model

### 2.1. Model of Uncertain Logistics Transportation System

In a green logistics system, a vehicle path usually has five basic components, namely transportation network, vehicle, logistics demand (hereinafter referred to as demand), renewable power generation, and warehouse.

1. Transportation network: This paper considers *𝕋* a discrete-time view. The duration of each time slot is *T*. Firstly, the logistics network is defined as a directed graph G(*V*, *V*), in which each vertex *i* ∈ *V* represents a point of interest (Point of interest, PoI); the PoI is composed of the intersection, the location of the freight car and the power source (charging pile and warehouse), and the place of delivery/distribution. Each side of (*i*, *j*) ∈ *V* is the road between these POIs and is influenced by the length *D*_*ij*_ and the estimated travel time *T*_*ij*_. Graph *G* can be established with two steps for any logistics network. First, sort out every PoI and set their coordinates in the figure. Then, the starting point and the ending point are connected by several edges, and each road needs to be reflected in the network.
2. Autonomous Vehicle: *V* is used to represent all logistics vehicles in the model, and every vehicle has its attributes, such as endurance mileage and logistics requirements. During the planning, each vehicle of *k* ∈ *V* starts the service request from the location *L*_*k*_^0^ ∈ *V* and stops at *L*_*k*_^*∗*^ ∈ *V*. Every vehicle has a battery which is ${\bar{E}}_{k}$ size. The initial energy of the battery is *E*_*k*_^0^. *E*_*k*,*ij*_ is the energy consumption of *K* to move over the road *(i, j*). The vehicle is charged at the charging point or warehouse at the rate of *R*_*k*_. Finally, the logistics transportation capacity of *K* is ${\bar{C}}_{k}$. The initial transportation requests is 𝒬_*k*_.
3. Logistics transportation request: The logistics request in the system is represented by the following parameters. 𝒬 is used to indicate the transportation request not received by any vehicle in the system. For any request $q\in 𝒬\cup \underset{k\in 𝒦}{\cup }{𝒬}_{k}$ in the model, *P*_*q*_^0^ and *P*_*q*_^*∗*^ are used to represent its extraction and delivery location, respectively. Before the time *T*_*q*_, the logistics transportation capacity *C*_*q*_ should be done.
4. Power generation or energy storage station: In the logistics system, vehicles will be charged at *d* ∈ *𝒟* energy storage station at *V*_*d*_, or *g* ∈ *𝒢* renewable power station located in *V*_*g*_. Vehicles can be charged free of charge from the energy storage station, which gets power directly from the grid. Each *g* can use Ω_*g*,*t*_ power to charge the vehicle at most in *t* period. The charging capacity of renewable energy is limited, and it is inefficient for cars to go back to a few parking lots. In the green logistics system and other logistics systems driven by electric vehicles, how to optimize the vehicle routing to meet the uncertain demand of logistics transportation under the premise of sufficient battery energy is a key problem.

RETRACTED

### 2.2. Online Route Selection Strategy

This paper mainly studies the online route selection strategy of uncertain green logistics system, which can guide vehicles through the city streets to fulfill the logistics requirements on the largest scale and charge fees according to needs. This can be modeled as an optimization problem. When the system status (such as logistics demand, charging pile power, traffic congestion, etc.) changes, the optimization problem is solved, and new vehicle routes are developed. *x*_*q*_^*k*^ is a binary indicator indicating whether the transportation request *q* ∈ 𝒬 is completed by vehicle *k*. *y*_*ij*_^*k*^ is also a binary indicator, indicating whether *k* will pass through the path (*i, j*). The transportation scheduling problem of uncertain green logistics system can be described as follows:

(1) $$\begin{array}{c} \text{minimize }C\sum_{k\in \kappa }\sum_{q\in Q}x_{q}^{k}-\sum_{k\in \kappa }\sum_{\left(i,j\right)\in \varepsilon }D_{ij}y_{ij}^{k}, \end{array}$$

where *C* is a large constant. The objective of this function is to maximize the amount of delivery logistics demand, minimize the distance traveled by the vehicles, and make a feasible path plan for all vehicles, which must comply with the system constraints. The constraints are as follows:

  The planned route must be connected
  Transportation needs should be met
  The logistics tasks must be completed within the specified time
  The load of each vehicle cannot exceed its logistics capacity
  The vehicle does not run out of power or overcharge
  During the charging process, the charging limit of the charging device needs to be observed

In order to model the objective problem as a constrained closed-form expression, it is necessary to use binary and continuous variables, and the problem becomes NP-hard. It can not effectively solve real scale problem examples. Therefore, this kind of problem formula can only make the offline path plan under the condition of given static system attributes, greatly affect the practicability of the logistics system, and can not solve the uncertain logistics transportation scheduling problem. In the uncertain logistics system, the submitted request can be modified, and new demand will be generated. The system needs to make corresponding adjustments to these dynamic changes in a short time.

RETRACTED

With the development of deep reinforcement learning technology, there are constantly new researches applied to the solution of combinatorial optimization problems. By adjusting the parameters of the deep reinforcement learning network, the solution effectively transfers the computational burden of the online solution development phase based on mathematical programming to the adjustment of offline parameters. Therefore, it can adapt to the dynamic changes of the system more quickly. The effect of the solution is very dependent on the neural network structure and the training process of the model parameters. This research adopts deep reinforcement learning to design a strategy that adapts to the uncertain green logistics system.

### 2.3. The Optimization Strategy

In the uncertain logistics transportation scheduling problem, given the transportation network *G*, the solution of this paper is to find a location of *π,* the sequence is called a journey, and each vehicle is constrained by constraints. The design of the transportation scheme requires that all pick-up/delivery places pass once in the shortest driving distance. If the vehicle needs to be charged, it can also pass through some charging facilities. These facilities and the places where it is required to pick-up/deliver are called stations. In each pair of connected stations, vehicles travel along the best route under the premise of meeting the constraints.

RETRACTED

In research involving neural network technology, an information center will be set to manage system status and other information. In the beginning, the dynamic state *S* of the current system will be sent to each vehicle through the information center. Then the logistics vehicle constructs a path map according to the current system state and transmits this result to the deep reinforcement learning network for the next step of itinerary planning. Finally, the information center collects the itinerary information of all logistics vehicles, and the logistics vehicles complete logistics tasks in accordance with the route map. The process is shown in Figure 1.

After each vehicle knows the current operating status of the system, it will first create a touring map and input it into the deep reinforcement learning network. Although you can choose to represent all nodes in the model in the deep reinforcement learning model when the number of nodes exceeds 100, the quality of the solution decreases, which corresponds to a minilogistics network. At the same time, the vehicles of the model are actually more sensitive to whether they will pick-up/send requests or stop charging as their next goal. On this basis, a method is proposed to simplify the traffic network to a smaller trip map of each vehicle.

Firstly, the possible stop locations of vehicle *k* are summarized. According to the model in Chapter 2, the vehicle will stop in the following positions:

1. Delivery place of on-board request: {*P*_*q*_^*∗*^*∣q* ∈ 𝒬_*k*_}。
2. Other request location: {*P*_*q*_^0^*∣q* ∈ 𝒬}
3. Delivery location of other requests: {*P*_*q*_^*∗*^*∣q* ∈ 𝒬}
4. All charging facilities: {*V*_*d*_*∣d* ∈ *𝒟*} ∪ {*V*_*g*_^*T*^*∣g* ∈ *𝒢*}
5. *K*'s destination: *L*_*k*_^*∗*^

Before the connection point *k* has no clear intention to stop, all other nodes in *𝒱* are only used as connection points. Therefore, all possible trips between these stations can be enumerated, and the trip graph of *k* is constructed as G_*k*_^*𝒮*^. In this figure, the nodes include the possible parking locations *L*_*k*_^0^ and the current vehicle locations summarized above. The edges constructed by these connection points are as follows:

  Connect *L*_*k*_^0^ to positions in groups 1, 2, and 4
  Connect all positions in groups 1–4
  Connect all positions in groups 1, 3 and 4 to *L*_*k*_^*∗*^

Figure 2 shows an example of how to create a path planning diagram under a given traffic network model. Finally, using the existing routing algorithms, such as *A*^*∗*^ search algorithms, the shortest path of each side (*i*, *j*) ∈ *ℰ*_*k*_^*𝒮*^ will be calculated. The distance, energy consumption, and estimated travel time of the path are named as *w*_*ij*_^*k*^, *u*_*ij*_^*k*^, *t*_*ii*_^*k*^.

RETRACTED

The main goal of the paper is to plan the minimum total travel distance by taking the system state and vehicle travel diagram as the input. This paper designs a pointer network model embedded in the structure diagram and designs the most reasonable path planning for each vehicle in the system.

Figure 3 consists of two parts: encoder and decoder. First of all, the encoder network on the left takes the system information, system status, and the path diagram of the planned part as input, and struct2vec to embed the system into the feature embedded signal of each node in *𝒱*_*k*_^*S*^. More specifically, struct2vec recursively extracts the characteristics of nodes according to the structural characteristics of its graph. Given a graph G_*k*_^*𝒮*^, the p-dimensional feature *μ*_*i*_^0^=0 for each *i* ∈ *𝒱*_*k*_^*𝒮*^ is initialized and embedded by struct2vec. Then update the corresponding embedded value by the following formula:

(2) $$\begin{array}{c} \mu_{i}^{r+1}\leftarrow f\left(x_{i},{\left\{\mu_{j}^{r}\right\}}_{j\in N\left(i\right)},{\left\{w_{ij}^{k}\right\}}_{j\in N\left(i\right)},{\left\{u_{ij}^{k}\right\}}_{j\in N\left(i\right)}\right.,\left.{\left\{t_{ij}^{k}\right\}}_{j\in N\left(i\right)};\Theta \right), \end{array}$$

where *r* is the number of iterations, *x*_*i*_ is the q-dimensional node feature of *i*, *𝒩*(*i*) is the neighbor of *i* in G_*k*_^*S*^, and *f*(·, Θ) is a parameterized nonlinear universal mapping. This update rule reflects that the basis of feature embedding comes from graph topology. Through *f*(·, Θ), the node characteristic *x*_*i*_ can spread to other neighbor nodes. The nonlinear propagation function is as follows:

(3) $$\begin{array}{c} \mu_{i}^{r+1}\leftarrow \text{ReLU}\left(\theta_{1}\sum_{j\in N\left(i\right)}\mu_{j}^{r}+\theta_{2}\sum_{j\in N\left(i\right)}\text{ReLU}\left(\theta_{3}w_{ij}^{k}\right)\right.+\theta_{4}\sum_{j\in N\left(i\right)}\text{ReLU}\left(\theta_{5}u_{ij}^{k}\right)\left.+\theta_{6}\sum_{j\in N\left(i\right)}\text{ReLU}\left(\theta_{7}t_{ij}^{k}\right)+\theta_{8}x_{i}\right), \end{array}$$

where *θ*_1_, *θ*_2_, *θ*_4_, *θ*_6_ ∈ *ℝ*^*p*×*p*^, *θ*_3_, *θ*_5_, *θ*_7_ ∈ *ℝ*^*p*^ and *θ*_8_ ∈ *ℝ*^*p*×*q*^ are system parameters. Re*LU*(*z*)=max{0, *z*} is the linear unit of unit level rectifier. The embedding computation of each node in *𝒱*_*k*_^*𝒮*^ is *r* iterations, where *R* is set to a small value in most studies, such as *R* *=* *4*. Then, the nodes are embedded in a recurrent neural network composed of LSTM (long-term memory) units, and a series of p-dimensional latent memory states {*C*_*i*_^enc ^ ∈ *ℝ*^*p*^}_*i*=1_^|*𝒱*_*k*_^*𝒮*^|^ are formed on the basis of receiving input data:

(4) $$\begin{array}{c} F_{i}=\sigma \left(W_{f}\cdot \left[h_{i-1},\mu_{i}^{R}\right]+b_{f}\right),\\ I_{i}=\sigma \left(W_{i}\cdot \left[h_{i-1},\mu_{i}^{R}\right]+b_{i}\right),\\ {\tilde{C}}_{i}=\tanh\left(W_{C}\cdot \left[h_{i-1},\mu_{i}^{R}\right]+b_{C}\right),\\ C_{i}^{\text{enc }}=F_{i}*C_{i-1}^{\text{enc }}+I_{i}*{\tilde{C}}_{i},\\ O_{i}=\sigma \left(W_{o}\cdot \left[h_{i-1},\mu_{i}^{R}\right]+b_{o}\right),\\ h_{i}=o_{i}*\;\tanh\left(C_{i}^{\text{enc }}\right). \end{array}$$

*σ*(*z*)=1/(1+*e*^−*z*^) is sigmoid function, *∗* is multiplication by element, *W*_*f*_, *W*_*i*_, *W*_*C*_, *W*_*o*_ is model weight parameter, *b*_*f*_, *b*_*i*_, *b*_*C*_, *b*_*o*_ is model deviation parameter. First, enter the embedding of *L*_*k*_^0^ into the network, and then enter the embedding of other sites in random order. Given that all nodes are embedded, the encoder encodes the graph structure and node characteristics as *C*_*𝒱*_*k*_^*𝒮*^_^enc^, which is input to the decoder as the initial unit storage state.

RETRACTED

Then, this article uses lstms to build the recurrent neural network model of the decoder in ptrnet. The encoder output is decoded to the station of the journey. The decoder maintains its potential memory state {*C*_*i*_^dec^ ∈ *ℝ*^*p*^}_*i*=1_^|*𝒱*_*k*_^*𝒮*^|^, which is calculated by formula (4). At first, a p-dimensional vector (g in Figure 3) as a trainable parameter of the entire network is inputted. Then the decoder constructs a complete process in an iterative manner. In the ith step, the memory state {*C*_*j*_^enc^}_*j*=1_^|*𝒱*_*k*_^*𝒮*^|^ used by the encoder and decoder, the current decoder state *C*_*i*_^dec^, and the constructed partial path *π*(<*i*) generate a distribution. The symbols used in this process are defined as follows:

(5) $$\begin{array}{c} a_{j}=\left\{\begin{array}{cc} v^{⊤}\cdot \;\tanh\left(W^{\text{enc}}C_{j}^{\text{enc}}+W^{\text{dec}}C_{i}^{\text{dec}}\right), & \text{ if vehicle }k\text{ can reach }j\text{ given }\pi \left(<i\right),\\ -\infty , & \text{otherwise,} \end{array}\right. \end{array}$$

(6) $$\begin{array}{c} \forall j=1,2,\ldots ,\left|V_{k}^{S}\right|,A\left({\left\{C_{j}^{\text{enc}}\right\}}_{j=1}^{\left|V_{k}^{S}\right|},C^{\text{dec}};W^{\text{enc}},W^{\text{dec}},v\right)≜\text{softmax}\left(a\right) \end{array}$$

where *v* ∈ *ℝ*^*p*^ is an observation vector and *W*^enc ^, *W*^dec ^ ∈ *ℝ*^*p*×*p*^ is an observation matrix. A (…) is the observation function, softmax (·) is the softmax function. In Figure 3, the larger arrow indicates the node with the highest probability. Therefore, our ptrnet specifies to visit the next station *π (i).* The probability is as follows:

(7) $$\begin{array}{c} p\left(\pi \left(i\right)|\pi \left(<i\right),S\right)≜A\left({\left\{C_{j}^{\text{enc}}\right\}}_{j=1}^{\left|V_{k}^{S}\right|},C^{\text{dec}}\right). \end{array}$$

This probability distribution represents that the decoder sees part of the path *π* (<*i*). The probability of system state *s* is given *π* (*i*). Randomly select all stops according to the probability distribution, expressed as *p*(*π*(*i*)*∣π*(<*i*), *𝒮*). The ergodic probability is as follows:

(8) $$\begin{array}{c} p\left(\pi |S\right)=\prod_{i=1}^{\left|V_{k}^{S}\right|}p\left(\pi \left(i\right)|\pi \left(<i\right),S\right). \end{array}$$

2.4. Solution of Uncertain Logistics Transportation Scheduling

This part proposes a scheme based on a deep reinforcement learning network. This scheme takes the characteristic values of the traffic network nodes as input and generates a complete traversal of these nodes through a good model parameter *π*. In this article, the purpose of introducing deep reinforcement learning networks is to reduce the computational burden brought by the increase in the number of vehicles. The supervised function can evaluate the cross-entropy between the output probability of the network and the optimal solution of the original problem. However, without a lot of calculation, it is difficult to get the optimal solution. In addition, due to the NP-hard nature of the vehicle routing problem, it takes a lot of computation time to construct a large training data set with an accurate solver, so this method is not practical. In this chapter, we use the forced learning technique of model free strategy to determine the model parameters, that is, the parameters in formula (3) *θ* Matrix, *W* and *B* matrix in formula (4) matrix in formula (5) *ν* and *W* matrix. Using symbols ϒ represents the collection of all parameters in the model.

RETRACTED

Firstly, an excitation function is designed for a single vehicle K, and then the function will help to adjust ϒ separately, So as to maximize the reward. Therefore, the training objective of the routing optimization problem should be used as the main consideration of the reward function, and the behavior that violates the constraint should be punished:

(9) $$\begin{array}{c} J\left(ϒ|S\right)=E_{\pi ∼p_{ϒ}\left(\cdot |S\right)}\left[O\left(\pi |S\right)-P\left(\pi |S\right)\right]. \end{array}$$

The overall training goal includes Monte Carlo sampling from the distribution:

(10) $$\begin{array}{c} J\left(ϒ\right)=E_{S∼P}J\left(ϒ|S\right). \end{array}$$

In formula (8) *O*(*π∣𝒮*) and *P*(*π∣𝒮*) are objective reward function and constraint penalty function, respectively.

(11) $$\begin{array}{c} O\left(\pi |S\right)=\sum_{q\in Q}x_{q}^{k}-C_{1}\sum_{\left(i,j\right)\in {Ε}_{\pi }\left(L_{k}^{*}\right)}w_{ij}^{k}, \end{array}$$

(12) $$\begin{array}{c} P\left(\pi |S\right)=C_{2}\sum_{q\in Q\cup Q_{k}}\max\left\{t_{P_{q}^{*},k}-T_{q},0\right\}n+C_{3}\sum_{i\in \pi }\max\left\{c_{i,k}-{\bar{C}}_{k},0\right\}+C_{4}\times c_{L_{k}^{*},k}n+C_{5}\sum_{i\in \pi }\max\left\{-e_{i,k},0\right\} \end{array}$$

Among them,

(13) $$\begin{array}{c} x_{q}^{k}=\left\{\begin{array}{cc} 1 & P_{q}^{*}\in \pi \\ 0 & \text{otherwise} \end{array},\;\forall q\in Q\right.,\\ {Ε}_{\pi }\left(i\right)=\left\{\left(\pi \left(j\right),\pi \left(j+1\right)\right)\left|j=1,2,\cdots ,\right|\left(\pi <i\right)|\right\},\\ t_{P_{q}^{*},k}=\sum_{\left(i,j\right)\in {Ε}_{\pi }\left(P_{q}^{*}\right)}t_{ij}^{k},\\ c_{i,k}=\sum_{j\in \pi \left(<i\right)}c_{j,k},\\ e_{i,k}=E_{k}^{0}-\sum_{\left(i,j\right)\in {Ε}_{\pi }\left(i\right)}u_{ij}^{k}+\eta R_{k}\times \left|\left\{i\in \pi \cap \left(\left\{V_{d}|d\in D\right\}\cup \left\{V_{g}|g\in G\right\}\right)\right\}\right|. \end{array}$$

*ℰ*_*π*_(*i*) is the journey *π* the edges connected to each other until they reach station *i,t*_*P*_*q*_^*∗*^,*k*_ is the time for *k* to reach delivery position *Q*, *c*_*i*,*k*_ is the used logical capacity of *k* at *i*, and *e*_*i*,*k*_ is the battery energy of *k* at *i*.

The gradient of formula (9) can be expressed by reinforcing the algorithm

(14) $$\begin{array}{c} \nabla_{\Upsilon }J\left(\Upsilon |S\right)=E_{\pi ∼p\Upsilon \left(\cdot |S\right)}\left[\left(O\left(\pi |S\right)-P\left(\pi |S\right)-b\left(S\right)\right)\times \nabla_{\Upsilon }\log\;p_{\Upsilon }\left(\pi |S\right)\right], \end{array}$$

where *b(s)* is an expected reward function estimated to be independent of *π* on the system state *S*, and it is also a baseline function. The gradient function can be approximated by the Monte Carlo sampling method as follows:

(15) $$\begin{array}{c} \nabla_{\Upsilon }J\left(Y\right)\approx \frac{1}{B}\overset{B}{\underset{i=1}{\sum }}\left[\left(O\left(\pi_{i}|S_{i}\right)-\right.\right.\left.P\left(\pi_{i}|S_{i}\right)-b\left(S_{i}\right)\right)\left.\times \nabla Y\;\log\;pY\left(\pi_{i}|S_{i}\right)\right], \end{array}$$

where *B* is the number of independent identically distributed samples in *S*_1_, *S*_2_,…, *S*_*B*_ ~ *P* and *π*_*i*_ ~ *p*_Υ_(·*|S*_*i*_).

The proposed ptrnet and critnet models are trained asynchronously by the asynchronous actor critical training method, and the parameters of the models are updated. During each iteration, the new path plan will be sampled from P first, and then ptrnet will be used for planning. The estimated reward values of these states are also generated by critnet, and then the gradient of ptrnet is calculated by formula (12). The mean square error of critnet can be expressed as (1/*B*)‖∑_*i*=1_^*B*^*b*_*i*_ − (*O*(*π*_*i*_*|𝒮*_*i*_) − *P*(*π*_*i*_*|𝒮*_*i*_))‖_2_^2^. Finally, we use Adam optimizer to adjust B on a small scale to update the model parameters. This completes an iteration of the training algorithm. When the parameters converge or reach the predefined maximum number of iterations, the algorithm stops.

RETRACTED

### 2.4. Experiment and Results

This article refers to the actual situation and sets a random value for the charging efficiency of each vehicle from 0.8 to 0.9 and sets a random initial charging state for each vehicle from 0.2 to 0.9. A random value between (0.3∼1.0) *D*_*ij*_ is set to the driving energy consumption of any road (*i*, *j*). The logistics capacity of each vehicle is randomly set between 50–100 units. Initially, 1 to 3 random requests are loaded on each vehicle as 𝒬_*k*_.

In addition, all needs are set in a randomly generated manner. In the logistics network, pick-up and receiving locations are randomly set from the existing POI, the deadline for delivery is a random value within 1 to 5 hours, and each demand is set from 5 Random values from units to 20 units and randomly assigned |*𝒱*|/4000 warehouses and |*𝒱*|/400 charging locations. When using DRL and CRITNET to train PTRNET, first extract the abstract logistics transportation network from the complete transportation network.

This article uses PyTorch to model the proposed neural network and simulates the process on several computing servers. In addition to two Intel Xeon e5-2683v4 CPUs, each server is equipped with 3.00 GHz and 128 GB of memory. Neural network calculations use NVIDIA GTX 1080ti GPU. Δ*t*=1min, {*C*_*i*_}_*i*=1_^7^={10^−4^, 10^−2^, 10^−2^, 10^−1^, 10^−1^, 10^−1^, 10^−2^},  *K*=2.

The greedy search method is labeled as DRL-greedy, and *M*∈{128, 1280, 12800} is labeled as DRL-sample @128, DRL-sample@1k, DRL-sample@13k Mark. This approach samples *M* candidate tours with respect to the probabilities developed by the stochastic policy *p*(*π*(*i*)*∣π*(<*i*), *𝒮*) is given in (7). Finally, we try sampling vehicular tours for one minute, and the best tour is labeled with DRL-sample@1 min. The intermediate solutions obtained by the mathematical program after searching for 1 min, 10 min, and 60 min are considered and labeled as MIP@1 min, MIP@10 min, and MIP@60 min. The results are shown in Table 1. In the test, the expression of the mathematical program, especially the mixed-integer program, is the same as the definition.

RETRACTED

At the same time, after searching for 1 minute, 10 minutes, and 60 minutes, the optimal solution is obtained from the evolutionary population, which is labeled as M-MOEA/D@1 min, M-MOEA/D@10 min, M-MOEA/D@60 min.

In Figure 4, the ratios of different path planning configurations to the optimal driving distance are sorted, and the performance comparison of manual transmission is illustrated in Figure 5.

Considering that logistics requests and available charging resources may change in real time and there are uncertainties, this paper randomly generates 100 cases. Each case contains 100 vehicles and 100 random initial requests and studies the impact of these uncertainties. The simulation result is shown in Figure 6. The figure shows the average number of requests that can be serviced and the average wait time before a request is responded. It can be seen from the table that although increasing the calculation time of the strategy may cause the system to generate more service requests, the positive benefits generated by the increased service requests may not be enough to offset the negative benefits generated by the longer request waiting time. Therefore, when the logistics system is in an uncertain state, the strategy proposed in this paper is better than the traditional logistics route planning strategy.

Next, use {*C*_*i*_}_*i*=1_^7^, {*C*_*i*_ × 0.1}_*i*=1_^7^, {*C*_*i*_ × 10}_*i*=1_^7^, {*C*_*i*_ × 100}_*i*=1_^7^ to train ptrnet and critnet, respectively, and the simulation results are shown in Figure 7. It is clear from the figure that {*C*_*i*_}_*i*=1_^7^ is the best performance set. This is because the number of local optima does not decrease, although a small {*C*_*i*_}_*i*=1_^7^ value will produce a smoother parameter search space.

In addition, the sensitivity of parameter *k* is tested, which controls the diversity of samples in the multisampling path construction scheme. Since K has nothing to do with the training process, the previously used fine-tuning model is used, and the influence of the K value on the proposed strategy is evaluated under different sampling configurations. Let *K* ∈ {1.2, 1.5, 2.0, 2.5, 3.0, 4.0}, and the result is shown in Figure 8. It is not difficult to conclude that the three configurations proposed in this article for the online logistics routing strategy, *K* = 2 is the best performance value of parameter *K*.

## 3. Conclusion

In this study, a new neural network combination optimization strategy based on deep reinforcement learning is proposed, which is used to develop the route planning of online traffic service vehicles, which is difficult to realize by traditional path generation algorithm with minimum computing time in a large network. In order to solve this problem, the deep reinforcement learning mechanism aims to improve the parameters of the neural network model. The scheme can improve the performance of the system effectively. The simulation results show that, under the limited computational time constraints, the strategy can develop excellent vehicle travel compared with the traditional strategy based on mathematical planning. Compared with traditional mathematical procedures, the algorithm proposed in this paper can reduce the driving distance by 60.71%. In addition, when the system is affected by factors such as logistics requirements and available charging resources, the quality of the solution will be further highlighted. Future work can use more advanced deep reinforcement learning network technology on the basis of this article to further realize the high performance of the system. At the same time, the research field of this article can be further expanded in the next stage to study the uncertain logistics and transportation problems in tram and nontram systems.

RETRACTED

## Figures and Tables

**Figure 1:** Flow chart of online path planning strategy for uncertain logistics system.

**Figure 2:** A tour graph creation.

**Figure 3:** Deep reinforcement learning network based on PTRNET and STRUCT2VEC.

**Figure 4:** Sorted driving distance ratios to optimality.

**Figure 5:** Performance comparison on manual speed changes.

**Figure 6:** Comparison of the performance of different online route planning schemes in uncertain logistics systems.

**Figure 7:** Sensitivity of parameter {*C*_*i*_}_*i*=1_^7^.

**Figure 8:** Sensitivity of parameter *K*.

**Table 1:** The performance of different strategies in uncertain logistics systems.

Strategy	Request served	Distance (km)	Computation
Optimal	200.00	3742.29	6.00 h
DRL-greedy	196.17	5855.68	0.51 s
DRL-sample@128	200.00	4612.84	3.96 s
DRL-sample@1k	200.00	4183.75	38.12 s
DRL-sample@13k	200.00	3966.61	379.44 s
DRL-sample@1 min	200.00	4139.84	60.00 s
MIP@ 1 min	200.00	10536.06	60.00 s
M-MOEA/D@ 1 min	198.03	4385.92	60.00 s
MIP@ 10 min	200.00	6150.25	600.00 s
M-MOEA/D@10 min	199.56	4004.19	600.00 s
MIP@60 min	200.00	3878.55	1.00 h
M-MOEA/D@60 min	200.00	3936.62	1.00 h

## Data Availability

Relevant data require the consent of all authors to be obtained.
